RETRACTED

# Efficacy of Chelerythrine Against Mono- and Dual-Species Biofilms of *Candida albicans* and *Staphylococcus aureus* and Its Properties of Inducing Hypha-to-Yeast Transition of *C. albicans*

**DOI:** 10.3390/jof6020045

**Published:** 2020-04-16

**Authors:** Weidong Qian, Jianing Zhang, Wenjing Wang, Miao Liu, Yuting Fu, Xiang Li, Ting Wang, Yongdong Li

**Affiliations:** 1 School of Food and Biological Engineering, Shaanxi University of Science and Technology, Xi’an 710021, China; qianweidong@sust.edu.cn (W.Q.); 1804070@sust.edu.cn (J.Z.); 201504040311@sust.edu.cn (W.W.); 1804065@sust.edu.cn (M.L.); 201504040401@sust.edu.cn (Y.F.); lixiang@sust.edu.cn (X.L.); 2 Ningbo Municipal Center for Disease Control and Prevention, Ningbo 315010, China

**Keywords:** *Candida albicans*, *Staphylococcus aureus*, chelerythrine, dual-species biofilm, antibiofilm activity

## Abstract

*Candida albicans* and *Staphylococcus aureus* specifically often resulted in biofilm-associated diseases, ranging from superficial mucosal to life-threatening systemic infections. Recent studies reported that chelerythrine displayed antimicrobial activities against a few microorganisms, but its effects on mono- and dual-species biofilms of *C. albicans* and *S. aureus* have never been reported. The purpose of this study was to evaluate the efficacy of chelerythrine against mono- and dual-species biofilms, and explore its effect on the hyphal growth and the hypha-to-yeast transition of *C. albicans*. The results showed that minimum inhibitory concentrations (MICs) and minimum biofilm inhibitory concentration (MBIC_90S_) of chelerythrine against planktonic cells of mono-species were 4 and 2 μg/mL, while the MIC and MBIC_90_ were 6 and 3 μg/mL for dual-species. Meanwhile, the decrease in three matrix component levels and tolerance to antibiotics of biofilms formed by mono- and dual-species exposed to chelerythrine were confirmed by a confocal laser scanning microscope, in conjugation with five fluorescent dyes and a gatifloxacin diffusion assay. Moreover, *C. albicans* and *S. aureus* mono-species showed a 96.4, and 92.3% reduction, respectively, in 24-h preformed biofilm biomass in the presence of 128 µg/mL of chelerythrine. Similarly, preformed (24 h) dual-species biofilm biomass also displayed a significant reduction (90.7%) when treated with 192 μg/mL chelerythrine. Chelerythrine inhibited hyphae formation of *C. albicans* at 4 μg/mL, and *C. albicans* in hypha-form can be converted into yeast-form at 8 μg/mL of chelerythrine. Therefore, chelerythrine shows promise as a potential antimicrobial and antibiofilm agent for clinical effective treatments of mono- and mixed-species and/or biofilm-associated infections.

RETRACTED

## 1. Introduction

*Candida* accounts for 70% to 90% of all human fungal infections and can be associated with devastating consequences, particularly in intensive care units where mortality rates reach 40% [1,2]. Oral candidiasis is one of the observed mostly human opportunistic fungal infections of the oral cavity, caused by an overgrowth of *Candida* species, the most common being *Candida albicans* [3]. *C. albicans*, a dimorphic fungal organism, is present primarily in the oral cavity in a non-pathogenic yeast state in about one half of healthy individuals, but, under nutrition-rich conditions, has the ability to switch to a disease-causing hyphae form [4]. Under poor oral health conditions, pathogens including methicillin resistant *Staphylococcus aureus* and *Pseudomonas aeruginosa* were easy to colonize in the oral cavity [5]. Oral microorganisms adhere to a surface and evolve to persist in the varying environments in protective biofilms [6]. Notably, in a diverse range of pathological niches, *C. albicans* often coexist with *S. aureus*, which are often co-isolated in cases of biofilm-associated infections, and have been implicated in blood, urinary tract, and burn wound infections, as well as infections of medical devices such as central venous catheters [7]. Specifically, *C. albicans* partners with *S. aureus* to enhance bacterial colonization and biofilm formation, where fungi can provide a scaffold for the biofilm formation of bacteria, thus allowing bacteria to survive in hostile environments or antibiotic treatments, and exacerbating mucosal tissue infection and destruction [8,9]. The complexity of polymicrobial biofilm-mediated infections presents an additional challenge to explore effective treatment strategies.

Biofilms are self-adhering communities of microorganisms embedded in a matrix of extracellular polymeric substances attached to an interface [10]. Biofilm formation involves several steps, namely the attachment to biotic or abiotic surfaces, maturation, and dispersal of mature biofilm and has long been recognized serve as a reservoir for pathogenic cells. Thus, biofilms can cause septicemia, and evolve into invasive systemic infections of organs and tissues [11]. The multifactorial nature of biofilms caused by mixed fungal-bacterial infections, along with the rapid emergence of antimicrobial resistance in pathogenic fungi and bacteria, imposes great challenges for the use of conventional antimicrobials, and further limits therapeutic options [12]. To prevent and address such stubborn infections caused by dual-species biofilm, effective anti-biofilm development and mature biofilm eradication agents are urgently needed. Nowadays, promising antimicrobials derived from natural extracts and isolated compounds from plants have attracted a lot of attention, due to their potential therapeutic value in various diseases and as a source of novel drugs.

RETRACTED

Chelerythrine, a benzo-c-phenanthridine alkaloid extracted from *Bocconia cordata*, has been utilized as a traditional medicine. Previous studies reported that chelerythrine exhibits various biological and pharmacological properties, including anti-cancer, anti-inflammatory, insecticide, anti-fibrosis activities, etc. [13,14]. A few recent studies reported antimicrobial activities of chelerythrine against *C. albicans*, *S. aureus*, *Escherichia coli*, and *Aeromonas hydrophila* [15,16,17,18]. However, the inhibitory and scavenging effects of chelerythrine against mono- and dual-species biofilms of *C. albicans* and *S. aureus*, as well as its effect on the hyphal growth and mature hypha switch of *C. albicans*, have yet to be fully investigated. Thus, the main purpose of this study was to evaluate the antibiofilm and mature biofilm eradication activities of chelerythrine against mono- and dual-species biofilms of *C. albicans* and *S. aureus*.

## 2. Materials and Methods

### 2.1. Reagents

Chelerythrine of HPLC grade was supplied by Chengdu Pulis biological science and Technology Co., Ltd. (Chengdu, China). Chelerythrine was dissolved in 1% dimethyl sulfoxide (DMSO, Sigma-Aldrich, St. Louis, MI, USA) and distilled water prior to use. SYTO 9, Film Tracer SYPRO Ruby, wheat germ agglutinin (WGA), propidium iodide (PI), and lipophilic membrane FM 4-64 dyes were purchased from Invitrogen (Thermo Fisher Scientific, Waltham, MA, USA). All other chemicals and solvents used were of analytical grade.

### 2.2. Bacterial Strains and Cultural Conditions

*Candida albicans* SC5314 and *S. aureus* ATCC25923 strains were employed and routinely grown in yeast peptone dextrose (YPD; 10 g/L of yeast extract, 20 g/L of peptone, and 20 g/L of glucose; Sigma-Aldrich, USA) and tryptic soy broth (TSB; Sigma-Aldrich, St. Louis, USA) medium under aerobic conditions at 37 °C for 18–24 h in a shaking incubator (180 rpm), respectively. The fungal and bacterial stocks were stored at –80 °C and supplemented with 25% glycerol (Sigma-Aldrich, St. Louis, USA) as a cryoprotectant. For mixed biofilm formation, *C. albicans* SC5314 and *S. aureus* ATCC25923 inoculum in saline solution at approximately 1 × 10^6^ CFU/mL were cultured on 1 cm × 1 cm glass coverslips in individual wells of a 24-well plate at 37 °C for 24 h in a shaking incubator (100 rpm).

### 2.3. Minimal Inhibitory Concentrations (MICs)

To determine the MICs of chelerythrine against *C. albicans* SC5314 and *S. aureus* ATCC25923, broth microdilution was performed according to the Clinical and Laboratory Standards Institute (CLSI) guidelines M27-A3 [19] and M7-M9 [20], respectively, with minor modifications. Briefly, overnight fungal and bacterial cultures were suspended in YPD and TSB at a final density of approximately 1 × 10^6^ colony forming unit (CFU) /mL, transferred into individual wells of the 96-well microtiter plate (Nunc, Copenhagen, Denmark), and then incubated with final concentrations of chelerythrine, ranging from 2 to 512 μg/mL. Fluconazole (64 μg/mL) and vancomycin (16 μg/mL) were employed as the positive control, while 1% DMSO was used as negative control group. After incubation at 37 °C for 24 h without shaking, the growth of *C. albicans* SC5314 and *S. aureus* ATCC25923 was examined by measuring the absorbance at 600 nm (OD_600_) using a Multiskan GO plate reader (Thermo Fisher Scientific, Waltham, MA, USA). The MIC was determined from independent triplicate assays and defined as the lowest concentration, at which microbial cell growth was not detected.

RETRACTED

### 2.4. Minimum Biofilm Inhibitory Concentrations (MBIC_90S_)

The minimum biofilm inhibitory concentration (MBIC_90S_), which is defined as the lowest concentration of antimicrobials that results in the inhibition of 90% biofilm formation, was quantified by the crystal violet (CV) assay and CFU enumeration. For the CV assay, overnight cultures of mono- and dual-species grown in YPD were firstly diluted to an inoculum dose of approximately 1 × 10^6^ CFU/mL. Then the dilution of *C. albicans* SC5314 and *S. aureus* ATCC25923 mono- and dual-species with a ratio of 1:1 was incubated in individual wells of a 96-well microtiter plate and treated with chelerythrine at 0, 1/16, 1/8, 1/4, 1/2, and MIC for 24 h. After incubation, the biofilms formed in individual wells were fixed with 200 μL of methanol after being gently washed three times with 5 mL phosphate buffered saline (PBS; 2.7 mM KCl, 1.5 mM KH_2_PO_4_, 136.9 mM NaCl, 8.9 mM Na_2_HPO_4_, pH 7.4). Then, the samples were stained with 200 μL of 0.1% crystal violet solution for 15 min. Followed by a 15 min inoculation, each well was washed with distilled water and added with 200 μL of acetic acid (33%, *v*/*v*), to dissociate the crystal violet attached to bacterial cell walls. For each sample, the absorbance at 570 nm was recorded by a microplate reader. Moreover, to calculate the number of viable fungal or bacterial cells, followed by treatment, the washed cells were then removed from each glass coverslip by washing with 1 mL of 10 mM PBS, then transferred into prelabeled microfuge tubes and sonicated for 10 min. The resulting cell suspensions of dual-species biofilms were diluted ten-fold and cultured on a sabouraud dextrose agar medium (SDA; Sigma-Aldrich, St. Louis, USA), supplemented with chloramphenicol (50 mg/L) (selective for *C. albicans*) and mannitol salt agar (MSA; Sigma-Aldrich, St. Louis, USA) (selective for *S. aureus*). Similarly, ten-fold dilutions of *C. albicans* and *S. aureus* biofilms were plated on SDA and MSA, respectively. After an additional 24 h incubation at 37 °C, the fungal and bacterial colonies were counted.

RETRACTED

### 2.5. Biofilm Inhibition Assay

The inhibitory effects of chelerythrine on the biofilm formation were observed by field emission scanning electron microscopy (FESEM; Nova Nano SEM-450, FEI, Hillsboro, OR, USA) and confocal laser scanning microscopy (CLSM; Zeiss LSM 880 with Airyscan), as described previously [21]. Approximately 1 × 10^6^ CFU/mL of mono-species and dual-species were cultured on the glass coverslips in individual wells of a 24-well microtiter plate, and treated with chelerythrine at 0, 1/8, 1/4, and 1/2 MIC at 37 °C for 24 h. For FESEM analysis, followed by treatment, the glass coverslips with biofilms were kept in sterile water containing 2.5% glutaraldehyde (*v*/*v*; Sigma-Aldrich, USA) at −4 °C for 2 h. Then, biofilms were rinsed three times with 10 mM PBS (pH 7.0) and dehydrated in water-alcohol solutions at various alcohol concentrations of 30%, 50%, 70%, 90%, and 100% for 10 min each. Finally, the resulting samples were characterized using a FESEM. Similarly, for CLSM analysis, the glass coverslips with biofilms were washed three times with 0.9% sodium chloride (NaCl) and incubated with 2.5 μM SYTO 9. After incubation at 25 °C for 15 min, the biofilms were examined by CLSM, where the fluorescence were measured at excitation/emission wavelengths of 485/542 nm for SYTO 9.

### 2.6. Biofilm Composition by CLSM

The composition changes of 24-h biofilms of mono- or dual-species were observed by CLSM. Briefly, approximately 1 × 10^6^ CFU/mL of mono-species and dual-species were cultured on the glass coverslip in each well of a 24-well microtiter plate and treated with chelerythrine of different concentrations (0, 1/8, 1/4, and 1/2 MIC) for 24 h at 37 °C. Then, the resulting samples were exposed to the following five types of dyes: (I) SYTO 9 dye, which stains nucleic acids; (II) Film Tracer SYPRO Ruby Biofilm Matrix stain, which labels most classes of proteins [22]; (III) WGA conjugated with Oregon Green, which stains N-acetyl-D-glucosamine residues [23]; (IV) PI dye that stains nucleic acids; (V) FM 4-64 dye, which stains lipophilic membrane. The fluorescence of dyes was measured using the following combination of excitation and emission wavelengths: 476 nm/500–520 nm for SYTO 9, 405 nm/655–755 nm for SYPRO Ruby, 459 nm/505–540 nm for WGA, 535 nm and 617–635 nm for PI, and for and 479nm/565–588 nm for FM 4-64, respectively. After each staining step, the biofilms were gently rinsed with 10 mM PBS. The biofilm images were acquired using a CLSM. Red/green fluorescence ratios to assess extracellular matrix components, including eDNA, proteins, and polysaccharides were measured on PI/SYTO 9, SYPRO Ruby/SYTO 9, and FM 4-64/WGA images, respectively, with KS 400 version 3.0 software (Carl Zeiss, Inc., Jena, Germany).

RETRACTED

### 2.7. Antibiotics Diffusion within Biofilms

To assess the diffusion capability of antibiotics in biofilms formed in the presence of chelerythrine, gatifoxacin diffusion within biofilms was measured based on its intrinsic fluorescence by CLSM [24]. Biofilms of mono- and dual-species were prepared in the same manner as described above on the glass coverslips placed inside the 24-well plate (Corning, NY, USA). The resulting biofilms were gently washed three times with 10 mM PBS, and a final concentration of 80 μg/mL gatifoxacin was added and further incubated for 5 h at 37 °C. Then, a final concentration of 3 μM SYTO 9 was added to visualize the gatifoxacin diffusion within biofilms. Followed by 15 min incubation, the samples were rinsed three times with 10 mM PBS to remove nonpenetrated gatifoxacin and observed using a CLSM. For an in-depth understanding of gatifloxacin diffusion scope and depth in biofilms, representative images in the z axis were obtained. At least three random fields were visualized for each biofilm.

### 2.8. Minimal Biofilm Eradication Concentration

To investigate the potential ability of chelerythrine to eradicate the preformed biofilms of mono- and dual-species, the preformed biofilm eradication assay was carried out in a 24-well microtiter plate, as previously described [25]. 24 h biofilms of mono-species and dual-species preformed on the glass coverslips in each well were treated with chelerythrine at different concentrations (0, 8, 16, and 32 MIC) for 5 h at 37 °C. Afterward, the biofilm was observed using a FESEM. Meanwhile, the biofilm biomass was measured by the crystal violet staining assay. Further, CFU recovery for viability was performed in treated biofilms as described above.

### 2.9. Effect of Chelerythrine on C. albicans Hyphal Growth and Mature Hyphae

Hyphal growth inhibition was examined according to hyphal length analysis. *Candida albicans* SC5314 was grown in YPD broth at 37 °C for 16 h in a shaking incubator at 180 rpm, washed twice with 10 mM PBS, and diluted to a concentration of approximately 1 × 10^6^ CFU/mL, using serum-free Roswell Park Memorial Institute 1640 medium (RPMI 1640; Invitrogen, Grand Island, NY, USA). For hyphal growth analysis, 100 µL of *C*. *albicans* cell dilution (approximately 1 × 10^8^ CFU/mL), 700 µL of fresh RPMI 1640 medium, and 200 µL of different concentrations of chelerythrine (0, 1/4, 1/2, and MIC) were mixed in each well of a 24-well culture plate, and cultured at 37 °C in 5% CO_2_ for 5 h. Thereafter, hyphae of *C. albicans* SC5314 were visualized using a FESEM. For mature hyphae analysis, 100 µL of *C. albicans* SC5314 cell dilution and 900 µL of fresh RPMI 1640 medium were mixed in each well of a 24-well culture plate, and cultured at 37 °C in 5% CO_2_ for 36 h. Subsequently, the resulting samples were treated with different concentrations of chelerythrine (0, 1/2, 1, and 2 MIC) for 4 h at 37 °C. Subsequently, the samples were observed by a FESEM.

RETRACTED

### 2.10. Statistical Analysis

All experiments were performed in triplicate. The data were expressed as mean values with the corresponding standard deviations (SD). Statistical analyses were performed with the statistical program SPSS software (SPSS 8.0 for Windows). Analysis of variance (ANOVA) was carried out to examine any significant differences (*p* ≤ 0.01).

## 3. Results

### 3.1. Minimum Inhibitory Concentrations (MIC_S_) and Minimum Biofilm Inhibitory Concentration (MBIC_90S_) of Chelerythrine against C. albicans and S. aureus

The MICs and MBIC_90S_ of chelerythrine against *C. albicans*, *S. aureus* mono- and dual-cultures were presented in Table 1. Chelerythrine displayed potent antibacterial activities to mono- and dual-cultures. The MICs and MBIC_90S_ of chelerythrine against *C. albicans* and *S. aureus* single cultures were 4 and 2 μg/mL. In addition, the MICs and MBIC_90S_ of chelerythrine against the mixed culture of *C. albicans* and *S. aureus* were 6 and 3 μg/mL.

### 3.2. Chelerythrine Decreased the Biofilm Formation of C. albicans and S. aureus Mono- and Dual-Species

The biofilm biomass of mono- and dual-species exposed to chelerythrine was measured using the crystal violet cell viability assay. As demonstrated in Figure 1A, the addition of chelerythrine reduced remarkably the biofilm biomass of the mono- and dual-species in a concentration-dependent manner. When *C. albicans* exposed to chelerythrine at the 1/8 MIC, there is a significant difference in the biofilm biomass between the treated and untreated group (*p* < 0.01). By contrast, the biofilm biomass of *S. aureus* mono- and dual-species in 1/4 MIC chelerythrine-treated groups displayed a significant difference, compared with the untreated group. The biofilm biomass of mono- and dual-species was further downregulated significantly (*p* < 0.001) after exposure to chelerythrine at 1/2 MIC or MIC, compared to the untreated control. The results showed that chelerythrine had an excellent inhibitory effect on the biofilm formation of *C. albicans* and *S. aureus* mono- and dual-species, and MBIC_90_ of chelerythrine against *C. albicans* and *S. aureus* mono-species biofilms were 2 μg/mL, while the MBIC_90_ of chelerythrine against dual-species biofilms was 3 μg/mL (Table 1). Moreover, after the biofilm formation of dual species for 24 h, the cell number of control samples was 9.2 log_10_ CFU/coverslip for *S. aureus* and 7.2 log_10_ CFU/coverslips for *C. albicans*, whereas overall a 6.5 to 4.1 log_10_ CFU/coverslips reduction was obtained for *S. aureus* and *C. albicans*, respectively, when treated with 1/4 MIC chelerythrine (Figure 1B). A similar trend was observed with a decline from 7.8 to 4.5 log_10_ CFU/coverslips for 1/4 MIC chelerythrine-treated *S. aureus* and *C. albicans* dual-species biofilm cells. For *C. albicans* and *S. aureus* mono- and dual-species biofilms tested, at 1/2 MIC chelerythrine concentrations, only 3.1 log_10_ CFU/coverslips or even less was observed. After treatment with MIC concentration, no survivors of either microbial cell were detected (Figure 1B).

RETRACTED

### 3.3. Sub-MIC Chelerythrine Changed the Biofilm Community Structure of C. albicans and S. aureus Mono- and Dual-Species

The basic biofilm structure of mono- and dual-species exposed to sub-MIC chelerythrine was analyzed by FESEM and CLSM. As demonstrated in Figure 2A, mono- and dual-species cells formed strong and sticky aggregates in the absence of chelerythrine. Especially, Figure 2A revealed also *S. aureus* to be distributed along the round *C. albicans* cells throughout the entire biofilm architecture, indicating the potentially synergistic relationship during polymicrobial growth. In contrast, subjecting mono- and dual-species cells to chelerythrine sub-MIC resulted in a less dense and loose biofilm network. Obviously, in the case of 1/2 MIC chelerythrine-treated group, the *C. albicans* mono- and dual-species biofilm structures were missing, and only individual cells can be viewed with disruption of the complex structure of the biofilms, but for *S. aureus* strains, distinct grape-like clusters appeared with less cell aggregations compared to the untreated group. In addition, in the treated group with chelerythrine at 1/8 MIC, biofilms of pure- and mixed-culture were generated by a dense and tight network of bacterial cells, except the treated groups had relatively low biofilm volumes.

We further examined the architecture of the biofilms in the presence or absence of chelerythrine by staining with SYTO 9 dyes to detect live cells using a CLSM. As shown in Figure 2B, a dense cluster composed largely of macrocolonies was present in the untreated *C. albicans* pure-culture group, while the biofilms cultivated in presence of chelerythrine appeared looser and more dispersed with the rise of the concentration used, suggesting that existing cell-cell adhesiveness inside the biofilm decreased over concentration. Similarly, in the absence of chelerythrine, a luxuriant homotypic biofilm was formed by *S. aureus* pure culture, whereas the less dense biofilm with the bubble-like structure was observed in the 1/2 MIC treated group, and less coverage gave way to loss of biofilm mass, similar to that delineated in the *C. albicans* biofilm. Similarly, in dual-species biofilms, mixed-culture biofilms treated with chelerythrine at 1/8 MIC presented a flake-like structure, with a significant increase in porosity, while the biofilm biomass remarkably decreased in the 1/2 MIC group, as compared with the 1/4 MIC group. These results showed chelerythrine at 1/2 MIC could effectively inhibit the biofilms formation *C. albicans* and *S. aureus* mono- and dual-species.

RETRACTED

### 3.4. eDNA Levels within S. aureus Mono-Species and C. albicans and S. aureus Dual-Species Biofilms Decreases in Response to Chelerythrine

To examine whether eDNA contributes to the observed decreased biofilm formation in response to chelerythrine treatment, CLSM image analyses were applied to investigate the in situ eDNA level, where eDNA was stained with a red fluorescent membrane impermeable DNA-binding stain PI, and SYTO 9, a green-fluorescent nucleic acid counterstain, was employed to stain cells of mono- and dual-species. As displayed in Figure 3A, in *S. aureus* mono-species, as well as *C. albicans* and *S. aureus* dual-species biofilms, the red labeling is more intense in a chelerythrine-free biofilm than in a biofilm formed in the presence of chelerythrine, revealing chelerythrine exposure reduced the eDNA quantity in a dose dependent manner. In contrast, in a *C. albicans* mono-species biofilm, the red fluorescence was less visible in the presence or absence of chelerythrine, indicating that the matrix of *C. albicans* biofilms contains a small amount of eDNA. Moreover, in the case of *S. aureus* mono-species, as well as *C. albicans* and *S. aureus* dual-species biofilms, some scattered yellow colorations caused by the superposition of the green (bacterial cells) and red (eDNA) fluorescence were observed in both the control and 1/8 MIC-treated groups, suggesting that eDNA was mostly localized inside these biofilms. To further evaluate the relative changes of eDNA within biofilms formed by mono- and dual-species of *C. albicans* and *S. aureus*, the relative intensity of eDNA fluorescence was calculated. As displayed in Figure 3B, the relative fluorescence intensities of eDNA in untreated *C. albicans* and *S. aureus* mono- and dual-species biofilms were significantly higher than those of biofilms of the 1/2 MIC-treated group (100%, 100%, and 100% versus 2.1% ± 1.0%, 3.3% ± 1.5%, and 7.2% ± 1.7%, respectively; *p* < 0.001). These results indicate that eDNA decrease contributes to a certain extent to chelerythrine-reduced biofilm formation by *S. aureus* mono-species and dual-species, while this situation was not suitable for *C. albicans* biofilms in response to chelerythrine.

RETRACTED

### 3.5. Chelerythrine Reduced the Biofilm Formation of C. albicans and S. aureus Mono- and Dual-Species by Mediating Extracellular Proteins Levels

To visualize the inhibitory effect of chelerythrine on *C. albicans* and *S. aureus* mono- and dual-species biofilms, the biofilm matrices were stained with two fluorescent dyes (SYPRO Ruby and STYO 9) and assessed by confocal laser scanning microscopy (CLSM). According to Figure 4A, chelerythrine significantly reduced *C. albicans* and *S. aureus* mono- and dual-species biofilm formation with a dose-related change. Interestingly, in *C. albicans* mono-species biofilms, a large number of extracellular proteins were seen in the control group, whereas at 1/4 MIC-chelerythrine treated group the protein contents were remarkably reduced, suggesting that extracellular proteins could play a role in *C. albicans* biofilm formation. Similarly, in *C. albicans* and *S. aureus* dual-species biofilms exposed to 1/4 MIC-chelerythrine, the density of extracellular proteins was remarkably reduced, compared with the untreated control. In contrast, in *S. aureus* mono-species biofilms, extracellular protein content of *S. aureus* biofilms decreased with the rise of chelerythrine concentration, but extracellular proteins were evenly embedded in the biofilm in the mosaic-like pattern. Imaging measurements demonstrated that the relative fluorescence intensities of proteins of untreated *C. albicans* and *S. aureus* mono- and dual-species biofilms were statistically higher than those of biofilms of 1/2 MIC treated group (100%, 100%, and 100% versus 2.2% ± 1.3%, 3.2% ± 1.6% and 0.6% ± 0.5%, respectively; *p* < 0.001) (Figure 4B). These results demonstrate that a decrease in the content of extracellular proteins contributed to a certain extent to chelerythrine-decreased biofilm formation by mono- and dual-species.

### 3.6. Chelerythrine Decreases the Biofilm Formation of C. albicans and S. aureus Mono- and Dual-Species by Mediating Extracellular Polysaccharides Levels

To assess the inhibitory effect of chelerythrine against *C. albicans* and *S. aureus* mono- dual-species biofilms, the biofilm matrix was stained with a combination of fluorescent stains wheat germ agglutinin and lipophilic membrane dye FM 4-64, and then evaluated by CLSM. As demonstrated in Figure 5A, in untreated *C. albicans* mono-species biofilms, CLSM images showed the green fluorescence occupied a significant part of the biovolume, suggesting a large number of extracellular polysaccharides in *C. albicans* biofilms. Interestingly, in the 1/8 MIC chelerythrine-treated *C. albicans* and *S. aureus* mono-species biofilms, a significant reduction in the content of the extracellular polysaccharides was observed, with a dose-independent manner. In contrast, in dual-species biofilms of *C. albicans* and *S. aureus*, extracellular polysaccharides levels decreased in a dose-dependent manner, and a large number of yellow fluorescence was distributed throughout the whole biofilm structure in the untreated group, indicating that mixed-culture contributed to extracellular polysaccharides production. Moreover, Figure 5B shows that the relative fluorescence intensities of polysaccharides in untreated *C. albicans* and *S. aureus* mono- and dual- species biofilms were significantly higher than those in biofilms of the 1/2 MIC-treated groups (100%, 100%, and 100% versus 0.8% ± 0.6%, 4.5% ± 1.6%, and 8.6% ± 1.6%, respectively; *p* < 0.001).

RETRACTED

### 3.7. Chelerythrine Treatment Reduces Mono- and Dual-Species Biofilms Tolerance to Gatifloxacin

Next, to assess the biofilms exposed to chelerythrine tolerance to antibiotics, gatifloxacin diffusion within mono- and dual-species biofilms was comparatively monitored using CLSM. As demonstrated in Figure 6, in untreated mono- and dual-species biofilms, we observed that gatifloxacin was confined to the outer periphery of the biofilm with minimal to no penetration into the biofilm. Also, under treatment with chelerythrine at 1/8 MIC conditions, a limited penetration of gatifloxacin into the mono- and dual-species biofilms was observed. In contrast, an increased penetration of gatifloxacin into the mono- and dual-species biofilms was found in the 1/4 MIC treatment group. Notably, under the concentration of chelerythrine at 1/2 MIC, it is obviously seen that gatifloxacin penetration was full within the mono- and dual-species biofilms, reaching the basal layers.

### 3.8. Chelerythrine Eradicates Efficiently Preformed Biofilms of C. albicans and S. aureus Mono- and Dual-Species

To confirm the biofilm eradication activity of chelerythrine, we evaluated the amount of and morphological changes to biofilms formed by mono- and dual-species influenced by exposure to chelerythrine at four sub-MIC concentrations, using the crystal violet staining assay and FESEM. As displayed in Figure 7A, the biofilm biomass of *C. albicans* and *S. aureus* mono-species was significantly reduced by treatment with chelerythrine at 16 MIC (*p* < 0.001), while a similar result was achieved at 32 MIC in dual-species group (*p* < 0.001). In addition, the removal potential of chelerythrine for mono- and dual-species mature biofilms was determined by FESEM. According to Figure 8, the eradication effect of biofilms enhanced as the chelerythrine concentration increased. Specifically, mature biofilms of *C. albicans* without chelerythrine treatment gave rise to dense aggregates, whereas >90% biofilms were eradicated when exposed to 16 or 32 MIC treatment. Similarly, treatment of *S. aureus* mono-species and dual-species biofilms with 32 MIC of chelerythrine resulted in almost complete degradation of biofilm architecture, and disaggregated the *C. albicans* and *S. aureus* cells in dual-species biofilms. The results were consistent with those obtained using the CVSA. Moreover, the results from CFU recovery displayed a remarkable decrease in *C. albicans* and *S. aureus* survival in a concentration-dependent manner when mono and mixed biofilms were treated with chelerythrine. Notably, 32 MIC chelerythrine treatment significantly diminished the ability of *C. albicans* and *S. aureus* mono- and dual-species biofilms to confer protection against viability of microbial cells (Figure 7B).

RETRACTED

### 3.9. Chelerythrine Inhibits the Hyphae Formation of C. albicans

The effect of chelerythrine on *C. albicans* hypha formation was further evaluated by incubating *C. albicans* in an RPMI-1640 medium supplemented with chelerythrine. As shown in Figure 9, massive *C. albicans* hyphae were observed in the untreated group, and *C. albicans* formed strong peripheral filaments. However, the growth of hyphae was markedly attenuated with the addition of chelerythrine at concentrations of 1/4 MIC and 1/2 MIC. Notably, hyphal formation was almost completely blocked by chelerythrine at the concentration of an MIC, where *C. albicans* cells were maintained as yeasts. These results reveal that chelerythrine inhibited the hypha formation in a concentration-dependent manner.

### 3.10. Chelerythrine Induce the Hypha-to-Yeast Transition in C. albicans

The effect of chelerythrine on the hypha-to-yeast transition was examined by FESEM. As shown in Figure 10, some untreated cells were found to have massive hyphae. In contrast, 1/2 MIC chelerythrine resulted in the formation of shorter hyphae, and a significant population of yeast forms was observed after treatment with MIC of chelerythrine for 5 h. Notably, at 2 MIC, chelerythrine treatment concentration cells were completely devoid of hyphae and remains in yeast form.

RETRACTED

## 4. Discussion

The mixed infection of *C. albicans* and *S. aureus* occurred frequently, which can lead to several diseases with a high mortality, rather than a single-species infection [26]. Synergistic interaction between *C. albicans* and *S. aureus* contributed to the development of polymicrobial biofilm communities, resulting in strong resistance to antibiotics, highlighting the need to find new antimicrobial agents [27]. In this study, we firstly examined the chelerythrine-mediated growth inhibition against mono- and dual-species planktic cells of *C. albicans* and *S. aureus*. The results showed MICs of chelerythrine were 4 μg/mL for both single *C. albicans* and *S. aureus* culture, while the MIC for a dual culture of *C. albicans* and *S. aureus* was 6 μg/mL. By contrast, He et al. showed that chelerythrine isolated from root of *Toddalia asiatica* (Linn) Lam exhibited a moderate growth-inhibitory effect against planktonic cells of *S. aureus* 25923, methicillin-resistant *S. aureus*, and extended spectrum β-lactamase *S. aureus*, and the MICs of chelerythrine against these three bacteria were all 156 μg/mL [13]. The data were higher than our results, which may be due to the purity of extracted chelerythrine extracted from *Toddalia asiatica* (Linn) Lam.

Moreover, biofilms protect embedded microbial cells against an in-principle adequate antimicrobials therapy, frequently resulting in treatment failure and relapsing infections. To further evaluate antibiofilm activities of chelerythrine against mono- and dual-species, a combination of CVSA, CFU enumeration, FESEM, and CLSM was employed. These results indicated that the MBIC_90S_ of chelerythrine for *C. albicans* and *S. aureus* mono- and dual-species were 2 and 3 μg/mL, respectively. Notably, the inhibitory concentration of chelerythrine against biofilm formation of mono- and dual-culture models of *C. albicans* and *S. aureus* was less than that of previous reports, where Shin and Eom reported that zerumbone remarkably inhibited mono- and dual-species biofilms formed by *C. albicans* and *S. aureus* at 64 μg/mL [28]. Similarly, She et al. showed that auranofin could effectively inhibit *S. aureus* and *C. albicans* mono- and dual-biofilm formation in vitro at 8 μg/mL [29]. Collectively, it can be concluded that chelerythrine had potent antibiofilm activities against a mono- and dual-culture of *C. albicans* and *S. aureus*. Interestingly, in contrast to the growth inhibitory potency against planktonic cells, the biofilm formation of *C. albicans* and *S. aureus* mono- and dual-species was more susceptible to chelerythrine with subminimal inhibitory concentrations (sub-MICs), respectively; however, biofilms formed over 24 h on a glass coverslips surface were more resistant to chelerythrine than were planktonic cells. The results are in agreement with previous studies, wherein sub-MICs of antimicrobial agents can suppress biofilm formation by affecting initial microbial adherence to surfaces [30,31]. It is important to highlight that chelerythrine displayed a significant inhibitory effect at the sub-MICs for biofilm growth, thus demonstrating its potential to minimize microbial resistance when combined with low-dose antimicrobials.

RETRACTED

Next, we further revealed the profile of extracellular proteins, polysaccharides, and eDNA of biofilms formed by mono- and dual-cultures of *C. albicans* and *S. aureus* after treatment with chelerythrine at sub-MIC. To this end, CLSM, in conjugation with five different fluorescent dyes, was applied to differentiate bacterial cells from proteins, polysaccharides, and eDNA within the biofilm matrix. The results confirmed that chelerythrine reduced biofilm formation by mediating mainly polysaccharides and eDNA levels for an *S. aureus* single culture, while for a *C. albicans* single culture, chelerythrine inhibited biofilm formation by decreasing mainly proteins and polysaccharides levels. These data were in line with previous reports that important components of *S. aureus* biofilm are extracellular polysaccharides and eDNA, while the *C. albicans* biofilm matrix is predominantly composed of proteins (55%), carbohydrates (25%), lipids (15%), and eDNA (5%) [32,33]. In agreement with these findings, for dual cultured of *C. albicans* and *S. aureus*, chelerythrine diminished biofilm formation by decreasing simultaneously extracellular proteins, polysaccharides, and eDNA levels in a dose-dependent manner. Interestingly, for chelerythrine-treated *C. albicans* mono-species and dual-species biofilms, the amount of eDNA was correlated positively with biofilm-forming capacity, suggesting that an abundant amount of eDNA was essential for the development of robust biofilms. In contrast, the importance of eDNA in biofilms may be overlooked in chelerythrine-reduced biofilm formation by *S. aureus* mono-species.

Meanwhile, hindered penetration of antibiotics through biofilms is one of the contributing factors to the remarkable increase in bacterial tolerance to antibiotics [34]. Here, we investigated the tolerance of biofilms of mono- and dual-culture of *C. albicans* and *S. aureus* after treatment with chelerythrine to antibiotics diffusion. To this end, gatifloxacin with intrinsic fluorescence in the range deep ultra-violet wavelength was employed to visualize the antibiotic diffusion through biofilm by CLSM. The results showed that gatifloxacin had minimal penetration into the matrix in the presence of chelerythrine at low concentration of 1/8 MIC, while gatifloxacin diffusion in both mono- and dual-species biofilms were increased significantly when exposed to chelerythrine at high concentrations of 1/2 MIC, revealing that the integrity of the mono- and dual-species biofilms was disrupted by chelerythrine, thereby enhancing the osmotic of biofilms.

RETRACTED

After verifying the antimicrobial and antibiofilm activities of chelerythrine, we investigated mature biofilm eradication activities of chelerythrine against mono- dual-microbial biofilms. It has been acknowledged that once the biofilm is well formed, the resistance to antimicrobials can be extremely increased. In the present study, chelerythrine could efficiently eradicate 96.4% and 92.3% 24 h mature biofilm formed by mono-cultures of *C. albicans* and *S. aureus* at concentrations of 128 μg/mL, and 90.7% 24-h mature biofilm of dual-culture at concentrations of 192 μg/mL, respectively. In contrast, Shin and Eom reported that treatment with 500 μg/mL of zerumbone resulted in a dramatic elimination of preformed *C. albicans* biofilm by 96.3% [28]. On the other hand, in the case of preformed *S. aureus*, dual-species biofilms were reduced by 49% and 39.4% at concentrations of 500 μg/mL, suggesting that chelerythrine was more effective in eradicating mono- and dual-species of *C. albicans* and *S. aureus* preformed biofilm than zerumbone.

Since hyphal growth plays an important role in *C. albicans* infection by mediating dissemination of *C. albicans* to the host tissues, the inhibition of *C. albicans* to hyphal growth forms is a significant finding [35]. Our results present that hyphal growth was remarkably inhibited at 4 μg/mL concentration of chelerythrine, showing a robust activity of chelerythrine against hyphal growth. In addition, the effect of chelerythrine on the mature hyphae of *C. albicans* was also tested. Hyphae of *C. albicans* in the presence of 4 μg/mL were shortened and majorly shifted to yeast state at 8 μg/mL concentration of chelerythrine used. A reason for shortening of *C. albicans* hyphae may be due to the reversible morphological plasticity between yeast and hyphal forms in response to chelerythrine. Similar results for reverse morphogenesis were observed with gymnemic acid, which transforms the hyphal cells of *C. albicans* into yeast cells [36].

RETRACTED

In addition, previous reports demonstrated that the anti-cancer effects of chelerythrine have been studied both in vitro and in vivo [37], thus attracting wide interest for its potential clinical applications. For example, NK109, a chelerythrine analogue, is in Phase 2 trial in Japan and 7-hydroxystaurosporine, a PKC inhibitor, in Phase 1 trials in the United States [38]. Further, Kosina et al. evaluated the effects of daily administration of the extract from *Macleya cordata* in the diet on the health status of swine. After 90 day administration the highest chelerythrine and sanguinarine (1:3) retention was detected in the gingiva (0.55 μg/g) and liver (0.15 μg/g), and treated animals did not demonstrate any results of hematological, biochemical, or histological assay different from controls [39]. Collectively, all of these results suggest that chelerythrine shows promise as a potential antimicrobial and antibiofilm agent for clinical effective treatments of mono- and mixed-species and/or biofilm-associated infections both in vitro and in vivo.

## Figures and Tables

**Figure 1:** Assessment of different concentrations of chelerythrine on *C. albicans* (CA) and *S. aureus* (SA) mono- and dual-species (SA+CA) biofilm biomass by crystal violet staining and cell enumeration by colony count. (**A**) The biofilm biomass was determined using the crystal violet staining assay. Values represent the means of triplicate measurements. (**B**) Biofilm production analysis was performed by cell enumeration (log_10_ CFU/coverslips). Bars represent the standard deviation (*n* = 3). * *p* < 0.05; ** *p* < 0.01; *** *p* < 0.001; NS, not significant.

**Figure 2:** Inhibitory effects of sub-MIC chelerythrine on *C. albicans* (CA) and *S. aureus* (SA) mono- and dual-culture (SA+CA) biofilms, shown in field emission scanning electron microscopy (FESEM, (**A**)) and confocal laser scanning microscopy images (CLSM, (**B**)). Scale bars represent 5 μm for FESEM and 10 μm for CLSM, respectively.

**Figure 3:** Effect of different concentrations of chelerythrine on the eDNA levels within *C. albicans* (CA) and *S. aureus* (SA) mono- and dual-species (SA+CA) biofilms by confocal laser scanning microscope. (**A**) eDNA was labelled with a red fluorescent membrane impermeable DNA-binding stain PI, and bacterial cells were stained with a green-fluorescent nucleic acid counterstain STYO 9. Scale bars represent 10 μm. (**B**) The relative fluorescence intensity of eDNA in biofilms of each treatment group was plotted against that in untreated group by measuring red fluorescence intensities using KS 400 version 3.0 software. Bars represent the standard deviation (*n* = 3). *** *p* < 0.001.

RETRACTED

**Figure 4:** Effect of different concentrations of chelerythrine on *C. albicans* (CA) and *S. aureus* (SA) mono- and dual-species (SA+CA) biofilm matrix structure. (**A**) Extracellular proteins were stained with a red fluorescent stain SYPRO Ruby, and *C. albicans* and *S. aureus* cells were stained with a green-fluorescent nucleic acid counterstain STYO 9. Scale bars represent 10 μm. (**B**) The relative fluorescence intensity of extracellular proteins in biofilms of each treatment group was plotted against that in untreated group by measuring red fluorescence intensities using KS 400 version 3.0 software. Bars represent the standard deviation (*n* = 3). *** *p* < 0.001.

**Figure 5:** Effects of different concentrations of chelerythrine on the levels of extracellular polysaccharides inside *C. albicans* (CA) and *S. aureus* (SA) mono- and dual-species (SA+CA) biofilms. (**A**) Extracellular polysaccharides were stained with a green fluorescent stain wheat germ agglutinin, and *C. albicans* and *S. aureus* cells were labelled with a red lipophilic membrane dye FM 4-64. Scale bars represent 10 μm. (**B**) The relative fluorescence intensity of extracellular polysaccharides in biofilms of each treatment group was plotted against that in untreated group by measuring green fluorescence ratios using KS 400 version 3.0 software. Bars represent the standard deviation (*n* = 3). *** *p* < 0.001.

**Figure 6:** Representative CLSM images assessing diffusion of gatifloxacin within *C. albicans* (CA) and *S. aureus* (SA) mono- and dual-species (SA+CA) biofilms formed in the presence of chelerythrine. After mono- and dual-species biofilms were grown for 24 h supplemented without or with chelerythrine of different concentrations, 0.4 mg/mL gatifloxacin was added into the medium. Following 5 h gatifloxacin diffusion, the biofilms were visualized using CLSM. Biofilms were stained with SYTO 9 for biofilms (green) and the intrinsic fluorescence of gatifloxacin (blue). Scale bars represent 10 μm.

**Figure 7:** Assessment of eradication effects of different concentrations of chelerythrine on *C. albicans* (CA) and *S. aureus* (SA) mono- and dual-species (SA+CA) mature biofilm biomass. (**A**) The biofilm biomass was assessed using crystal violet staining assay. (**B**) Mature mono and mixed species biofilms were treated with different concentrations of chelerythrine, and fungal or bacterial cell viability was examined by CFU recovery. Values represent the means of triplicate measurements. Bars represent the standard deviation (*n* = 3). * *p* < 0.05; ** *p* < 0.01; *** *p* < 0.001; NS, not significant.

**Figure 8:** Scanning electron microscopy images of *C. albicans* (CA) and *S. aureus* (SA) mono- and dual-species (SA+CA) mature biofilms after treatment with four MIC-fold concentrations of chelerythrine. Each field of vision was magnified 10,000×. Scale bars represent 5 μm.

RETRACTED

**Figure 9:** The effect of chelerythrine on the hyphal growth of *C. albicans*. *Candida albicans* cells were grown in an RPMI-1640 medium at the indicated concentration of chelerythrine at 37 °C for 24 h. Each field of vision was magnified 5000×. Scale bars represent 10 μm.

**Figure 10:** The effect of chelerythrine on *C. albicans* mature hyphae. *Candida albicans* mature hypha were formed in RPMI-1640 for 24 h and treated with indicated concentrations of chelerythrine for 5 h at 37 °C. Each field of vision was magnified 5000×. Scale bars represent 10 μm.

**Table 1:** Minimum Inhibitory Concentrations (MIC)s and Minimum Biofilm Inhibitory Concentration (MBIC_90S_) of chelerythrine against mono- and dual-species planktonic cells of *Candida albicans* and *Staphylococcus aureus*.

Strain	MIC_S_ (μg/mL)	MBIC_90S_ (μg/mL)
*Candida albicans* SC5314	4	2
*Staphylococcus aureus* ATCC25923	4	2
Dual species	6	3
